# Application of Microfluidics in Immunoassay: Recent Advancements

**DOI:** 10.1155/2021/2959843

**Published:** 2021-07-15

**Authors:** Yuxing Shi, Peng Ye, Kuojun Yang, Jie Meng, Jiuchuan Guo, Zhixiang Pan, Qiaoge Bayin, Wenhao Zhao

**Affiliations:** School of Automation Engineering, University of Electronic Science and Technology of China, Chengdu 611731, China

## Abstract

In recent years, point-of-care testing has played an important role in immunoassay, biochemical analysis, and molecular diagnosis, especially in low-resource settings. Among various point-of-care-testing platforms, microfluidic chips have many outstanding advantages. Microfluidic chip applies the technology of miniaturizing conventional laboratory which enables the whole biochemical process including reagent loading, reaction, separation, and detection on the microchip. As a result, microfluidic platform has become a hotspot of research in the fields of food safety, health care, and environmental monitoring in the past few decades. Here, the state-of-the-art application of microfluidics in immunoassay in the past decade will be reviewed. According to different driving forces of fluid, microfluidic platform is divided into two parts: passive manipulation and active manipulation. In passive manipulation, we focus on the capillary-driven microfluidics, while in active manipulation, we introduce pressure microfluidics, centrifugal microfluidics, electric microfluidics, optofluidics, magnetic microfluidics, and digital microfluidics. Additionally, within the introduction of each platform, innovation of the methods used and their corresponding performance improvement will be discussed. Ultimately, the shortcomings of different platforms and approaches for improvement will be proposed.

## 1. Introduction

In recent years, point-of-care testing has become a hot topic in scientific research, including research on immunoassay, biochemical analysis, and molecular diagnosis. The reason is that point-of-care-testing can not only achieve less reagent consumption but also provide a strong guarantee for the early diagnosis of diseases. Among various point-of-care-testing platforms, the microfluidic chip is a new trend of innovation development.

Microfluidic chip utilizes the technology of miniaturizing conventional laboratory based on fabrication of the microchannel network, which enables the whole biochemical process including reagent loading, reaction, separation, and detection on the microchip. The common features of microfluidic platforms include fluid transport, fluid metering, fluid valving, fluid mixing, and reagents incubation [1, 2]. These microfluidic chips have the following advantages. First, the amount of reagent consumption can be dramatically decreased through scaling down the assay volume. Second, the surface force (capillary force, etc.) plays a dominant role in the motion of liquid as the characteristic scale decreases, which makes it possible for passive liquid propulsion such as capillary test strips. Third, laminar flow with a low Reynolds number can produce a stable liquid-liquid interface, paving the way for higher sensitivity [2].

Immunoassay is a biochemical test that measures the concentration of an analyte (mostly protein) in a solution by using an antibody or antigen [3]. The common immunoassay methods are as follows: enzyme-linked immunosorbent assays (ELISA), radioimmunoassays, fluorescence immunoassays, chemiluminescence, and so on. Although immunoassay has become a common analysis method, the traditional immunoassay needs complex operation steps and huge experimental equipment, which affects the promotion of immunoassay in POCT. However, the combination of immunoassay and microfluidic can greatly improve the shortcomings of traditional immunoassay.

In recent years, many scientific researchers have explored and studied the improvement of immunoassay performance when detecting analytes in blood or other secretory fluids. In the meanwhile, tens of thousands of researchers have published their works on the application of microfluidics in immunoassay. Among their attempt for improvement, some focus on the simplification of steps, some on the integration of systems, and some on the improvement of sensitivity. Researchers are committed to developing a complete microfluidic platform for ideal integration and good packaging without losing sensitivity.

So far, there have been many reviews of the application of microfluidics in different aspects [4], as well as reviews specifically of certain microfluidics, such as the biomedical analysis of centrifugal microfluidics [5]; however, there has not been any review of different microfluidic platforms specifically for immunoassay applications. Besides, the development and innovation of microfluidic immunoassay have been changing rapidly. For instance, an ultra-low-cost paper centrifugal operating system that can be operated manually was invented in 2017 [6], and Tan et al. developed a reusable optofluidic point-of-care testing platform for the sensitive detection of biomarkers with simple procedures [7]. Therefore, a review about immunoassay application on various microfluidics is urgent for researchers who study POCT in areas with limited resources.

In this review, the latest application of microfluidics in immunoassay in the past decade will be reviewed. According to different driving forces of fluid, microfluidic platform is divided into two parts: passive manipulation and active manipulation (shown in Figure 1). In passive manipulation, we focus on the capillary-driven microfluidics, while in active manipulation, we introduce pressure microfluidics, centrifugal microfluidics, electric microfluidics, optofluidics, magnetic microfluidics, and digital microfluidics. Additionally, within the introduction of each platform, innovation of the methods used and their corresponding performance improvement will be discussed. Finally, the shortcomings of different platforms and approaches for improvement will be proposed.

## 2. Application of the Passive Microfluidic System in Immunoassays

Over the years, a great number of developments of passively driven microfluidic lab on chip have emerged. Microfluidics is usually driven and propelled without the external actuator. According to the forces used, the passive microfluidic technology can be divided into capillarity-driven, surface tension, gravity-driven flow, and so on [8].

The passive microfluidic system has many unique advantages. Firstly, it is easy to be fabricated. Secondly, less expertise is needed as there is no requirement for trained operators. Thirdly, compared to active microfluidic systems, it costs less as no external power is required [8]. Recently, many researchers have combined immunoassays with a passive microfluidic system and have made great progress such as better valve control [9], unprecedented level of integration [10], and high sensitivity [11].

These automated passive microfluidic immunoassay systems perform equally or even better compared to those precise laboratory experiments. Therefore, the system is a promising tool for regions with limited resources.  Table 1 summarizes some classical passive microfluidic immunoassay systems.

### 2.1. Capillary-Driven Microfluidics

From the Laplace capillary pressure formula (*р*∼2 *λ*/*R*, *λ* is the surface tension of the liquid and *R* is the capillary radius), we can know that when the capillary radius becomes smaller, the capillary pressure will increase. Capillary pressure is a power source, which can drive the flow without the input of external energy. When applied to microfluidic chip, it can remarkably reduce the volume of the driving device. The typical capillary-driven microfluidic immunoassay platform is listed in Table 1.

#### 2.1.1. System Integration, Portability, and Step Simplification of Capillary Microfluidic Immunoassay

Some researchers have made great efforts on the system integration, portability, and operation step simplification of capillary microfluidic immunoassay.

In 2017, as is shown in Figure 2, Li et al. developed a way to control capillary-driven fluid transport in paper-based microfluidic devices with the use of a movable valve, which made up the shortcoming of applying mechanical means to control the capillary-driven fluid movement. In this way, the fluid could be controlled freely without timing setting. This device was used for the detection of carcinoembryonic antigen (CEA) which yielded a limit of detection (LOD) of 0.3 ng/mL within 60 min [9].

Avoiding high system complexity, such as multistep operation, is the key to achieving the efficient use of microfluidic devices. In 2018, a simple capillary-driven microfluidic platform without washing step was reported. Epifania et al. realized single-step mode of operation for the detection of mycotoxin by using integrated microbeads. The LOD was 1.7 ng/mL [10]. Based on the previous simplification of the operation steps, in 2019, Yakoh et al. introduced a 3D capillary-driven paper-based sequential microfluidic device for the detection of *α*-Feto Protein (AFP). With the help of an origami folding paper (oPAD) and a movable reagent-stored pad (rPAD), this device not only avoided the complicated steps in the experimental operation but also gained an LOD of 0.63 ng/mL within 30 min [12]. In addition, the simplification of the steps and the integration of the system are often inseparable. In 2020, Dogan et al. developed a passive microfluidic device to detect *Escherichia coli* (*E. coli*) and *Salmonella enteritidis* (*S. enteritidis*) with the LOD of 5 and 3 cfu/mL within 60 min. This device adopted the fluorescence technique with magnetic nanoparticles (MNPs) to separate target bacteria and quantum dots. Pipetting the samples and reagents is the only required step, which greatly facilitates portability [13].

#### 2.1.2. Sensitivity Enhancement of Capillary Microfluidic Immunoassay

Hard work has been done by researchers to shorten the detection time and increase the sensitivity of capillary microfluidic immunoassay system.

In 2013, Hu et al. developed a portable flow-through fluorescent immunoassay lab-on-a-chip device using ZnO nanorod-decorated glass capillaries for the detection of three biomarkers. As shown in Figure 3(a), the use of zinc oxide (ZnO) nanorods increased surface area for high-density probe attachment meanwhile amplified the fluorescent signal. This device gained an LOD of 1 ng/mL, 5 ng/mL, and 5 ng/mL for prostate-specific antigen (PSA), a-fetoprotein (AFP), and carcinoembryonic antigen (CEA), respectively, in 30 min [14]. The effective immobilization of antibodies is a thorny problem in improving sensitivity. In 2018, Pham et al. introduced a way to immobilize antibodies in which rabbit IgG antibodies were captured on the beads functionalized with capture antibodies and bound by detection antibodies (dAbs) conjugated to gold nanoparticles. An LOD of 24.6 ng/mL for rabbit IgG was achieved in 20 min [15]. Similarly, in 2019, Pham et al. presented immunogold silver staining assays on capillary-driven microfluidics for the detection of malaria antigens, and the combination of sandwich immunoassays with electroless silver staining yielded an LOD of 6 ng/mL in 20 min [16]. In 2020, Hemmig et al. transposed lateral flow immunoassays to capillary-driven microfluidics by using self-coalescence modules and capillary assembled receptor carriers (as shown in Figure 3(b)). They immobilized receptors inside closed microfluidic devices in 30 s, and the whole detection time was less than 25 min with the LOD of 4 ng/mL [11]. In 2020, Lin et al. developed a capillary-driven microfluidic immunoassay system in glass capillaries of 1 mm internal diameter. The surface-to-volume ratio of the reaction was increased by this strategy, and the reaction time was shortened to 45 min with an LOD of 0.46 ng/ml for anti-p53 autoantibody detection [17].

### 2.2. Gravity-Driven Microfluidics

The advantage of gravity-driven microfluidics is similar to that of capillary-driven microfluidics. The independence of additional driving force makes it cheap to fabricate and significantly improves the system integration.

As for the sensitivity improvement, Kadimisetty et al. developed a 3D-printed supercapacitor-powered electrochemiluminescent (ECL) protein immunoassay with high sensitivity and low cost in 2015. The reagents' propelling and washing were realized by the gravity flow used in hand screen-printed carbon sensors. Detection limits of prostate-specific antigen (PSA), prostate-specific membrane antigen (PSMA), and platelet factor 4 (PF-4) were 300 fg/mL, 535 fg/mL, and 420 fg/mL, respectively [18]. In order to quickly measure the kinetics of single islet secretion in a nonprofessional laboratory, in 2017, Schrell et al. introduced online fluorescence anisotropy immunoassay for monitoring insulin secretion from islets of Langerhans. This system used a gravity-based system to carry out experiments on different glucose levels, which yielded an LOD of 4 nM [19]. Apart from the sensitivity improvement, the stability and repeatability of the system are also very essential. In 2019, Li et al. presented a way for quantitative detection of digoxin with the use of small-molecule immunoassay in a recyclable gravity-driven microfluidic device. The high stability and reproducibility were attributed to a two-signal-mode small-molecule immunoassay with an internal reference included. What is more, they could recycle the beads when the beads were retained in the G-Chip simply by incubating the chip with the dissociation buffer. As a result, this device could be recycled for at least 50 times without any complicated operations [20]. In 2019, Wu et al. presented a gravity-driven chemiluminescence paper-based microfluidic device for the detection of chromium (III) (Cr(III)) for the first time. With the use of paper which eliminates the complicated external fluid control equipment, the LOD reached 0.0245 mg/L but the cost of the device further decreased [21]. As a kind of modern portable electronic product, smartphone enables the information processing ability for detection of analyte by exerting its inner functions such as image processing. In 2017, Shang et al. developed a paper-based microfluidic dot ELISA system with smartphone for the detection of influenza A. The image was captured by the smartphone camera and was processed by its own intelligent algorithm developed by Java [22].

## 3. Application of the Active Microfluidic System in Immunoassays

In recent years, many active microfluidic systems have appeared in the market. Active microfluidics aims at precisely controlling the reaction chamber in the chip through the external instrument. The control of liquid reaction position, the real-time monitor of the flow state of liquid in the chip, and the quantitative control of the volume of reaction sample make the sample participate in the immune reaction quantitatively, thus achieving real and accurate control.

According to different external driving forces, active microfluidics can be divided into centrifugal microfluidics, magnetic microfluidics, electrophoretic microfluidics, digital microfluidics, optofluidics, and so on.

### 3.1. Centrifugal Microfluidic System in Immunoassays

Centrifugal microfluidics is a kind of microfluidics system which uses centrifugal force as the driving force of liquid flow to realize the detection and analysis of reagents.

Centrifugal microfluidics embraces many advantages. First, as shown in Figure 4, centrifugal force exists in every corner of the disk, so that the transportation of liquid becomes simple and efficient. Second, the physical and chemical properties of analytes, such as pH value and viscosity, have little influence on the centrifugal microfluidic control panel, which is good news for blood and other analytical samples. Third, centrifugal microfluidics can achieve a high degree of integration [24, 25]. The whole experimental process including sample pretreatment, sample mixing, sequential liquid loading, and valve control can be realized on a single disk. The typical centrifugal microfluidic immunoassay platforms are listed in Table 2.

#### 3.1.1. Improvement in the Aspects of Mixing Efficiency, Step Simplification, Stability, and Accuracy

In 2009, Yusoff et al. developed a lab-on-a-disk with applied centrifugal force employed as a potential microfluidic platform to reduce the assay time by effectively mixing and separating liquid in the ELISA assay [23]. Compared to the conventional microwell for the detection of dengue NS1, the reagents consumption reduced from 760 *μ*l to 75 *μ*l. In order to further promote the mixing performance of the system, in 2011, Lee et al. used silica beads with a larger mass and a laser-irradiated ferrowax microvalve (LIFM, an active valve based on the phase transition of ferrowax) to complete the detection of 6 different analytes in 22 min (as shown in Figure 5(a)) [26]. In the same year, Noroozi et al. presented a multiplexed immunoassay system based upon reciprocating centrifugal microfluidics. The key to the design of the microfluidic control panel was the reciprocating structure (as shown in Figure 5(b)). The centrifugal acceleration acting on the disk firstly generated and stored the pneumatic energy and then released the pneumatic energy by reducing the centrifugal acceleration, resulting in the reversal of the liquid flow direction. This reciprocating structure was combined with the pneumatic valve, thus greatly improving the mixing efficiency [27]. Similarly, in 2013, Kim et al. introduced a flow-enhanced electrochemical immunosensor for the detection of c-reactive protein (CRP) on centrifugal microfluidic platforms. Compared with the optical density method, 17-times improvement was achieved with an LOD of 4.9 pg/mL [28].

In addition to the improvement of mixing efficiency, the stability and accuracy of centrifugal microfluidic devices are also crucial. In 2018, Arjmand et al. designed and fabricated a centrifugal microfluidic device with a septum valve for the detection of hemoglobin A1c in human whole blood. The entry and exit of reagents were precisely controlled by this novel valve. Within 8 minutes, 14 samples of human whole blood HbA1c were monitored, and the standard deviation was ±0.36%, indicating that the system was very stable [29].

On the basis of effective mixing and system stability, scientists are committed to the development of multiplexed centrifugal microfluidic disk to obtain high-throughput detection. In 2018, Miyazaki et al. presented a label-free, spatially multiplexed SPR detection of immunoassays on a highly integrated centrifugal lab-on-a-disc platform (as shown in Figure 6). There were two valves, the event-triggered valve and the centrifuge-pneumatic siphon valve (CPSV), which enabled the fluidic process including integration and parallelization of plasma extraction, metering, and all the following steps of the multiplexing immunoassays detection. The LOD of the immunoglobulin G (IgG) was 19.8 *μ*g/mL within 1 hour [30]. Similarly, in 2018, Phaneuf et al. developed a disposable disc with automatic aliquoting inlets paired with a noncontact heating system. This device was used for the detection of three enterotoxins (cholera toxin, staphylococcal enterotoxin B, and Shiga-like toxin 1) simultaneously. The experiment was completed within 1 hour with an LOD of 1.35–5.50 ng/mL [31]. In 2019, as shown in Figure 7(a), Mandi et al. used fixed elastic reversible (FER, in which sealing pressure was controlled through adjusting the engraving depth of the valve seat) valves and tunable elastic reversible (TER, in which the sealing pressure depended on how deep the plastic screw goes into the valve seat) valves to develop a microfluidic device with peptide microarrays for automated multiplexed detection of five different proteins within 40 min [32].

Traditional immunoassay usually needs complex and professional operation steps as well as professional training personnel to operate. Centrifugal microfluidic immunoassay platform, as a modern medical device for point-of-care-testing, is urgent for steps simplification. In 2018, Gao et al. presented a centrifugal microfluidic device for the detection of carcinoembryonic antigen in clinical serum samples. As the effects of the medium density, rotation speed, and spin duration were investigated, the device realized a washing-free assay with an LOD of 0.7 ng/mL [33]. Similarly, in 2020, as shown in Figure 7(b), Lin et al. developed a centrifugal device for washing-free detection of procalcitonin (PCT). This washing-free centrifugal microchip fluorescence immunoassay employed centrifugation step (15 s) to remove residual liquids and minimize nonspecific adsorption so that the washing step could be eliminated. The experiment was completed in 10 min with an LOD of 0.10 ng/mL [34].

#### 3.1.2. Improvement in the Aspects of Automation, Integration, and Miniaturization

As a potential development object of POCT, the centrifugal microfluidic immunoassay platform is supposed to be more automated, integrated, and miniaturized. However, complicated operation steps, large equipment volume, and complex external equipment are all obstacles to further promotion of such platforms.

In 2012, Ukita et al. developed a stacked centrifugal microfluidic device with three-dimensional microchannel networks and multifunctional capillary bundle structures for the detection of anti-mouse IgG. The device with multiple layers of disk-like chips greatly facilitated the integration and miniaturization of the system. The experiment was completed in 25 min with an LOD of 1 ng/Ml [35]. In order to improve the system integration by innovating the valve control, in 2017, as shown in Figure 8, Wang et al. applied an actuator which was composed of a flyball governor and a group of spring plungers to form an integrated immunoassay system for the detection of rabbit anti-mouse IgG. Four sequential valves and one inward pump were integrated to gain an LOD of 20 ng/mL [36]. Similarly, in 2017, Lutz et al. introduced a fully integrated microfluidic platform for the sensitive detection of Troponin T and NT-proBNP. A disk-like microfluidic disposable cartridge containing all required dried and liquid reagents was an important part of the system. The LOD was 7.55 ng/L and 16.566 ng/L for Troponin T and NT-proBNP, respectively [37]. Both switching the rotation frequency [43–46] and mechanically controlling the opening and closing of the valve [47, 48] to realize the sequential loading of the flow would definitely increase the cost and size of the microsystem. In 2018, Okamoto and Ukita developed an automatic microfluidic enzyme-linked immunosorbent assay based on CLOCK-controlled autonomous centrifugal microfluidics for the detection of human albumin. As shown in Figure 9(a), this CLOCK-controlled system realized the automatic operation of the ELISA assay at a steady rotational frequency, which eliminated the use of a huge external speed controller. The experiment was completed within 18 min with an LOD of 0.516 ng/mL [38]. As large-scale production was unsuitable for the aforementioned ELISA system using PDMS as a substrate, based on the CLOCK-controlled system, Abe et al. further increased the integration of the platform. They developed a lab in a bento box which was an autonomous centrifugal microfluidic system for the detection of mouse IgG. As shown in Figure 9(b), a small centrifugal microfluidic device driver (bento box) and a centrifugal microfluidic device made of polypropylene and fabricated by injection molding formed the system. The experiment was completed within 12 min with an LOD of 0.32 ng/mL [39].

As for the improvements in automation, in 2015, Czilwik et al. executed a magnetic chemiluminescent immunoassay for human C-reactive protein on the centrifugal microfluidics platform. All the processing steps were performed in the automated system with the aid of a set of stationary magnets and a microfluidic polymer disposable. The experiment was completed within 25 min with an LOD of 1.5 ng/mL [40]. In 2017, Zhao et al. conducted c-reactive protein and interleukin 6 microfluidic immunoassays with on-chip prestored reagents and centrifugo-pneumatic liquid control. Prestorage and release of liquid reagents were achieved with the use of stick-pack technology. The automation of the whole system completely depended on frequency switching without external operation. The LOD was 1.0 ng/mL and 64 pg/mL for CRP and IL-6, respectively [41]. To acquire higher integration, in 2020, an enhanced centrifugation-assisted lateral flow immunoassay for the point-of-care detection of prostate-specific antigen was conducted by Shen et al. As shown in Figure 9(c), the whole operation steps of the experiment including sample preparation, flow actuation, and washing were automatically operated on the centrifugal platform with the combination of a nitrocellulose membrane inserted into the centrifugal microfluidic system and the integrated microfluidic device itself. The whole process was completed in 15 min with an LOD of 0.028 ng/mL, which was 21.4-times of that of lateral flow immunoassay (LFIA) [42].

### 3.2. Magnetic Microfluidic System in Immunoassays

#### 3.2.1. Magnetic Nondigital Microfluidic System in Immunoassays

Magnetic force and microfluidics are no longer new concepts, but the combination of the two has been a new research hotspot in recent years. Different from electrokinetic microfluidics, magnetic microfluidics is less affected by surface charge, ion concentration, temperature, and pH. Similarly, magnetic manipulation does not require direct contact with fluid which is a good choice of external pumping force [49].

Magnetic force can manipulate not only magnetic objects and particles in microchannels but also nonmagnetic objects. Therefore, magnetic microfluidics has made great contributions to the development of innovative valves in microfluidics, the development of solid carriers for biological reactions in microchannels, and the capture of target analytes [50].

In this section, the related applications of magnetic microfluidics in recent five years will be described. In these applications, magnetic microfluidics will assist the realization of liquid pumping, mixing, valve control, and other functions. At the end of this section, a new magnetic-related digital microfluidic will be introduced. The typical magnetic microfluidic immunoassay platforms are listed in Table 3.

With the help of magnetic force, the detection accuracy of microfluidic immunoassay system has been significantly improved. Aiming at removing the limitation of the analysis of single analyte based on the discrimination between bound and unbound magnetic nanoparticles, in 2005, Kim and Park conducted a magnetic force-based multiplexed microfluidic immunoassay using superparamagnetic nanoparticles, in which the specific applied magnetic field only moved the microbeads conjugated with superparamagnetic nanoparticles by analytes consequently to the high gradient magnetic fields. The experiment was completed within 35 min with an LOD of 244 pg/mL and 15.6 ng/mL for rabbit IgG and mouse IgG measured, respectively [51]. In order to overcome the shortcomings of traditional tools such as centrifuge tube in the capture process of complex three-dimensional microstructure, a microchip-based immunomagnetic detection of circulating tumor cells was developed by Hoshino et al. in 2011 in which the effective capture of labeled cells was achieved by the combination of the thin, flat dimension of the microchannel, and the sharp magnetic field gradient (as shown in Figure 10(a)). A comparable capture rate was obtained by 25% less magnetic particles compared to the conventional system [52]. To overcome the limitation for the detection of small molecules at low concentrations by conventional surface plasmon resonance (SPR) techniques, in 2014, Guo figured out an amplification approach with the combination of magnetic Fe_3_O_4_@Au nanoparticles (GMNPs) and a magnetic field for an SPR immunoassay. This LOD of human interleukin 17A was 0.05 ng/mL, which was lower than that by using aptamer-Au NPs conjugates [53]. The photoelectrochemical (PEC) sensing method is a novel technique. However, the actual application of PEC immunoassay is still restricted because the photoactive material of the sensor mainly depends on photoactive metal semiconductor. In 2017, Lin et al. developed a new PEC immunoassay system in which the whole experiment was performed on anti-AFB1 antibody-modified magnetic beads by using glucose oxidase- (GOx-) labeled AFB1-bovine serum albumin (AFB1-BSA) (as shown in Figure 10(b)). The LOD was 2.1 pg/mL with a dynamic working range from 0.01 to 20 ng/mL under optimal conditions [54]. In 2017, Sharafeldin et al. employed a novel composite of Fe_3_O_4_ nanoparticles loaded onto graphene oxide (GO) nanosheets (Fe_3_O_4_@GO) to realize a mediator-free detection of prostate-specific antigen (PSA) and prostate-specific membrane antigen (PSMA). The experiment was completed with an LOD of 15 fg/mL and 4.8 fg/mL [55]. Similarly, in 2018, Zhou et al. created a novel magnetic PEC system by using reduced graphene oxide functionalized BiFeO_3_ (rGO-BiFeO_3_) as the photoactive material for the detection of PSA. An ultralow LOD of 0.31 pg/mL was acquired in the experiment [56]. In order to avoid unwanted magnetic capture of the magnetic particles caused by remanence when using magnetic materials in the microfluidic immunoassay system, Rabehi et al. presented a magnetic frequency mixing technique with a set of miniaturized planar coils for the highly sensitive detection of superparamagnetic beads. The experiment was completed with an LOD of 15 *μ*g/mL without any shielding [57]. In 2019, Guo et al. conducted a magnetic quantum dot nanobead-based fluorescent immunochromatographic assay for the detection and quantification of aflatoxin B1 (AFB1). In the experiment, magnetic fluorescent beads (MFBs) displayed ca. 226-fold stronger fluorescence emission with the use of octadecylamine-coated CdSe/ZnS QDs (OC-QDs) and oleic acid-modified iron oxide nanoparticles (OAIONPs) capsulated into two polymer matrixes. An LOD of 3 pg/mL was achieved in the experiment [58]. With the rapid development of smartphone, the combination of smartphone and microfluidic immunoassay has been frequently explored in recent years. In 2019, Zheng et al. used nanoparticle aggregation and smartphone as an imaging tool for the highly sensitive detection of *Escherichia coli* O157 : H7 in a microfluidic immunoassay system. The smartphone imaging tool measured the color to quantify the bacteria with an LOD of 50 cfu/mL [59]. With the development of space technology, the highly sensitive visual detection of proteins in space is becoming more and more important. In 2020, Li et al. developed a chip-based scientific payload technology for visual detection of interleukin- (IL-) 6 in spaceflight in which they successfully gained immunoaffinity enrichment and highly sensitive detection by using superparamagnetic immunoassay particles (as shown in Figure 10(c)). An LOD of 250 pg/mL was gained in the experiment [60].

Apart from the improvement of the detection accuracy, in a POCT system, the systematization of the system, the rapidity of the experiment, and the simplification of the steps are equally of significance. In 2016, with the aim of overcoming the limitation of conventional ELISA for difficulty in integrating with low-volume bioreactors, as shown in Figure 11(a), Riahi et al. used disposable magnetic microbeads for immobilization and integrated microvalves in the device to realize the automation of steps such as bead loading, binding, and washing [61]. In the same year, Uddin et al. applied an on-disc magnetic field-assisted incubation protocol [76] to realize the automation of assay steps which yielded an LOD of 25 pM within 15 min 30 s [62]. To decrease the complexity of the assay which used multiwavelength or light scattering for quantification, in 2017, Soares et al. developed a novel integrated device with manually operated magnetic valves for the detection of ochratoxin A (OTA), aflatoxin B1 (AFB1), and deoxynivalenol (DON). The LOD of these three kinds of fungi was 100 ng/mL, 100 ng/mL, and 3 ng/mL, respectively [63]. In some conventional optimized magneto-immunoassays [77, 78], fluorescent [79] and magnetic beads (MB) incubation are conveyed under agitation and MB washings rely on magnets, which hinder the integration with a low-cost POC device. In 2020, as shown in Figure 11(b), Ruiz-Vega et al. presented a POCT device for sensitive malaria detection in whole blood based on magnetic beads, Poly-HRP, and microfluidic paper electrodes in which the washing step, detection step, and filtration step were all conducted in an integrated disposable paper microfluidic device [64]. SERS-based competitive immunoassays based on conventional microtubes and magnetic bars are faced with a problem of requirement for manual washing steps. In 2016, Gao et al. used magnetic immunocomplexes trapped by yoke-type solenoids embedded within the device for the direct SERS signals measurement [65]. Similarly, for SERS, in order to reduce the complex photolithography process for fabricating the SERS substrate, in 2017, Yap et al. made use of bifunctional plasmonic magnetic nanoparticles to integrate micromixing and SERS detection. This method not only increased the integration of the system but also reduced the assay time from 4 h to 80 min [66]. For further improving the integration of the POCT immunoassay system for the detection of HIV-1 p24 antigen, in 2020, as shown in Figure 11(c), Liu et al. presented a fully integrated multicolor immunosensor in which all the immunoreaction steps and the gold nanorod based assay were integrated into a single chip. Through moving magnetic beads to different aqueous phases, the experiment was completed with an LOD of 0.5 ng/mL for the detection of HIV-1 p24 antigen [67].

In terms of multiplex and high-throughput detection, in 2011, Tang et al. used biofunctionalized magnetic graphene nanosheets (MGO) as immunosensing probes and multifunctional nanogold hollow microspheres (GHS) as distinguishable signal tags. This method realized a multiplexing immunoassay detection for highly sensitive detection of carcinoembryonic (CEA) and alpha-fetoprotein (AFP) [68]. Similarly, for cancer biomarker multiplexing detection, in 2012, Malhotra et al. presented an ultrasensitive detection of interleukin 6 (IL-6), IL-8, and vascular endothelial growth factor (VEGF) in the clinic with the use of a nanostructured microfluidic array in which the beads were magnetically separated into the array when they finished the capturing of the proteins and the washing step. A superlow LOD of 5–50 fg/mL was obtained [69]. In 2020, as shown in Figure 12(a), Armbrecht et al. conducted the sensitivity detection and quantification of protein secretion from circulating tumor cells in microfluidic chambers. The multiplexing detection was achieved by using the barcoded magnetic beads which were capable of CTC profiling in future work [71]. For the heart disease biomarkers detection, in 2019, chemiluminescence immunoassays for simultaneous detection of copeptin, heart-type fatty acid-binding protein (h-FABP), and cardiac troponin I (cTnI) based on magnetic carbon composites and the three-dimensional microfluidic paper-based device were presented by Yang et al. And in the detection, Co2+/N-(aminobutyl)-N-(ethylisoluminol) (ABEI) functionalized magnetic carbon composite (Co2+-ABEI-Fe_3_O_4_@ void@C) was used as an interface. The LOD of the experiment was 0.40 pg/mL, 0.32 pg/mL, and 0.50 pg/mL, respectively [70]. In 2020, as shown in Figure 12(b), a novel magnetic microfluidic sensor with nanostar antennas was developed for the multiplexing detection of cardiac troponin I (cTnI) and neuropeptide Y (NPY) in which the LOD of 0.0055 ng/ml and 0.12 ng/ml was yielded, respectively [72].

One of the most important preconditions for POCT to be popularized is the low cost of mass production. In 2015, an integrated microfluidic system for measurement of glycated hemoglobin levels by using an aptamer-antibody assay on magnetic beads was developed by Chang et al. The reduction of cost of the assay was owing to the elimination of the use of the first antibody. To the best of our knowledge, this was the first time that aptamer was used as a test for glycated hemoglobin [73]. The use of magnetic pump can greatly increase the cost of POCT product design. In 2019, Gao et al. developed an SERS-based immunoassay in which a pump-free microfluidic device was created as a detection platform [74]. In 2019, Coarsey et al. developed a flow-free magnetic actuation platform for sensitive detection of HIV-1, the p24 capsid antigen in which syringe pumps or other peripherals to maintain the flow were not required. In this way, the cost of the device was greatly reduced without the loss of accuracy [75].

#### 3.2.2. Magnetic Digital Microfluidic System in Immunoassays

Another microfluidic model developed using magnetic force is the concept of droplet-based microfluidics, also known as the “digital microfluidics” [80]. Because of the high surface area volume ratio of microfluidics, the experimental reagents can be greatly saved by controlling and operating the droplets resulted from liquid surface tension [81].

Droplet preparation can be divided into “active” and “passive” methods. The former requires some external energy for droplet manipulation, such as electric, magnetic, or centrifugal force, while the latter only needs several simple microfluidic chip structures to produce droplets. Therefore, the “passive” method is more widely used. There are three common “passive” droplet preparation methods: T-junction, flow focusing, and coflow.

The basic mechanism of digital microfluidics is similar to the traditional methods, but the volume of liquid involved is much smaller, and the process is highly automated [82]. Digital microfluidic devices usually use magnetic particles to separate and extract analytes [83]. For example, a droplet can pass through an electrode array in a digital microfluidic device to a magnetic electrode, where the magnetic particles are functionalized so that they can bind to the target analyte [84]. The application of this kind of immunoassay has been outstanding in recent years.

In 2008, Sista et al. conducted heterogeneous immunoassays using magnetic beads on a digital microfluidic platform to solve the problem of clogging of channels in the conventional assay. The experiment was completed in 7 min for the detection of human insulin and interleukin6 (IL-6) [85]. In 2012, Ng et al. presented a digital microfluidic (DMF) magnetic separation for particle-based immunoassay, in which they eliminated the use of oil carrier fluid (for droplet movement) to form a particle-based immunoassay for the first time. The volume of reagents used in the new method was reduced by 100 times and the time was shortened by 10 times compared to the conventional method [86]. In order to eliminate the requirement of a complicated solenoid fabrication procedure and precise control of the magnetic field, in 2016, Gao et al. developed a wash-free magnetic immunoassay of the PSA cancer marker using SERS and droplet microfluidics in which the magnetic bar was used for segregation of the free and bound SERS tags. This method could achieve rapid detection without washing [87]. Similarly in wash-free, in 2018, Gao et al. conducted a multiplexing immunoassay of dual prostate cancer markers using an SERS-based microdroplet channel in which they adopted a permanent magnet to align the magnetic immunocomplexes on one side of the channel [88]. The complex and intricate electrode fabrication hinders the development of digital microfluidic. In 2018, as shown in Figure 13, a SERS-based immunoassay with DMF was employed by Wang et al. to form a highly sensitive detection of the H5N1 virus [89]. For shorter detection time and less manual operation, in 2019, Coudron et al. made use of the advantages of the full magnetic separation process with antibody-bound microbeads to form a fully integrated digital microfluidics platform for automated immunoassay with minimal washing steps. Therefore, the experiment was completed within 6–10 min with high sensitivity [90]. To overcome the lack of separation of the microparticles from the whole blood based on the existing microparticles, in 2020, Cowell et al. developed a sensitive and multiplexing detection of interleukin-6 with the use of electrically distinct hydrogel beads in which highly monodisperse populations of magnetic hydrogel beads (MHBs) were produced by droplet microfluidic synthesis [91]. For system miniaturization, in 2020, Guan et al. presented an open surface droplet microfluidic magnetosensor which applied a miniaturized multifunctional 3D printing optosensing accessory for immunoassay incubation [92].

### 3.3. Electrophoresis Microfluidic System in Immunoassays

Electrophoresis on microfluidic chips (EMC) depends on the induction of detectable differences in migration behavior between charged species induced by applied electric field. Under the action of electric field, charged particles move towards the opposite electrode. This kind of technology has been studied by many researchers because of its less reagent consumption, lower cost, shorter detection time, and higher integration [93].

The common electrophoretic microfluidics is as follows: capillary electrophoresis microfluidics, gel electrophoresis microfluidics, dielectrophoresis microfluidics, and field (electric) flow fractionation [93]. This section focuses on the improvement of different aspects of electrophoresis microfluidics platforms.

Some researchers have made efforts in mixing efficiency. In 2017, Hu et al. conducted simulation analysis on improving microfluidic heterogeneous immunoassay with the use of induced charge electroosmosis on a floating gate. They used the induced charge electroosmotic (ICEO) convection in a low concentration suspension to improve the transportation efficiency of biomolecules. Compared to the conventional pressure-driven flow system, the binding efficiency increased by 4 times [94]. In order to further solve the problem of the slow diffusive mass transfer of the analyte to the binding surface, in 2020, Ge et al. used the electroconvective stirring driven by external AC electric fields to greatly enhance the binding reaction efficiency of the antigens towards the antibodies. In this experiment, the phenomenon of induced charge electroosmosis in a rotating electric field (ROT-ICEO) was the core innovation to improve the reaction efficiency [95]. Similarly, in 2020, Selmi and Belmabrouk applied the AC electroosmosis (ACEO) to produce swirling structures in the fluid through which the transportation efficiency of the antigen to the immobilized antibodies was greatly enhanced [96].

A few researchers have made remarkable progress in detection accuracy and sensitivity. In 2017, a nanoplasmofluidic device integrated with microelectrodes combined with AC electroosmosis-enhanced localized surface plasmon resonance (ACE-LSPR) biofunctional nanoparticle imaging technology was used for the sensitive detection of IL-1*β*, which yielded 158.5 fg/mL for spiked samples in PBS and 1 pg/mL for diluted human serum [97]. As AC electrothermal (ACET) does not function effectively in electrophoresis or electroosmosis, in 2017, Yang et al. employed the AC electrokinetics (ACEK) effects to perform the reagent and analyte delivery, incubation, and flushing. The experiment time was shortened from 30 minutes to about 1 minute with an LOD of 0.1 *μ*g/mL for the detection of *Mycobacterium avium* subsp. paratuberculosis (MAP) [98]. Similarly, in 2018, an integrated immunoaffinity extraction and separation device for the detection of Preterm birth (PTB) biomarker was developed, and in this device, the immunoaffinity extraction protocols were combined with microchip electrophoresis. The experiment was completed within 30 min with an LOD of 2 ug/mL [99]. In order to further improve the detection performance of the system, in 2019, as shown in Figure 14, Xie et al. developed an aptamer-based assay with the combination of a catalytic hybrid assembly and a microfluidic chip electrophoresis format. The LOD of alpha-fetoprotein, carbohydrate antigen 125, and carcinoembryonic antigen were, respectively, 0.1 pg/mL, 0.2 pg/mL, and 0.15 pg/mL, which reached a new height of sensitivity [100].

Researchers have done hard work in multiplexing, step simplification, and automation. Aiming at overcoming the shortcomings of traditional Western blotting, such as long time, cumbersome manual steps, poor repeatability, and large sample consumption, Jin et al. improved the method to achieve multiplexed detection. Separated tracks were used for the deposit of multiple injections from the same sample. The experiment with high throughput, high automation, and high sensitivity was completed in 8 min [102]. Similarly, in 2020, Arvin et al. carried out a fast immunoassay for microfluidic Western blotting by direct deposition of reagents onto the capture membrane. Proteins separated by microchip electrophoresis can be trapped on the membrane by dragging the membrane which greatly reduces the separation and transfer time of Western blotting to a few minutes (within 1 hour) [101]. To make up for the shortcoming of the most methodologies and procedures used for the detection of glycomarkers, that is, too many experienced techniques and trained steps, in 2016, Lesur et al. conducted an experiment in which the addition of lectin in the electrophoresis buffer was used in CGE to enable lectin affinity electrophoresis, and the liquid-phase binding assay facilitated the formation of the microfluidic-based automated immunoanalyzer [103]. In terms of dielectrophoresis, in 2011, Yang et al. presented a high-throughput system assisted with dielectrophoresis for multiplexed detection of IL-2, IL-6, IL-10, and TNF-*α*. In this experiment, a nonuniform electric field was employed to induce dielectrophoresis (DEP) force for the manipulation of the beads. More than 70% of the target molecules were captured in this experiment [104].

### 3.4. Optofluidic System in Immunoassays

As a new technical research field in the recent ten years, optofluidics is very suitable for biochemical analysis of small volume analytes (Figure 15 illustrates the structure and principle of typical optofluidic devices). Because optofluidics is the integration of photonics and microfluidics, many optical properties including refractive index, fluorescence, and Raman scattering can be used alone or in combination to sense signals. Combined with traditional immunoassay methods, optical microfluidics can render accurate control, manipulation, and real-time monitoring of the analysis process [105]. For example, optofluidic fluorescence detection was used to improve the light-fluorophore interaction to obtain a lower limit of detection, and optofluidic SERS can enhance the number of target analyte molecules to get better performance. All in all, photohydrodynamics is a very promising research field. This chapter mainly focuses on the application of immunoassay in optofluidics and the clarification of the mechanism of performance improvement in various aspects of the immunoassay process.

In recent years, there have been many explorations in improving the detection sensitivity. In 2018, Liang et al. developed a fiber light-coupled optofluidic waveguide (FLOW) immunosensor for the sensitive detection of p53 protein. In this experiment, they enlarged the shape factor *R* to strengthen the evanescent-wave interaction, and they increased the sensitivity with the combination of the proposed FLOW immunosensor and flowing microfluid. The LOD of the experiment was 10 fg/mL [106]. To further enhance the sensitivity of turbidimetric immunoassay, in 2019, Yang et al. presented a novel optofluidic laser TIIA (OFL-TIIA) for the detection of IgG. The novelty of this device was the increase of the loss induced by antigen-antibody complexes via the amplification effect. The reason was that the immunoreaction in the OFL-TIIA method occurred in a laser cavity. Due to this method, an outstanding limit of detection (LOD) (1.8 × 10^−10^ g/L) was achieved [107]. Similarly, in 2020, a nanomaterial-enhanced fiber optofluidic laser biosensor for the detection of enzyme horseradish peroxidase (HRP) was created. The Au nanorods and SiO_2_ nanoparticles were selected as demonstrative models to be coated onto the surface of thin-wall hollow fiber so that they obtained high sensitivity as nanomaterials owned a high surface-to-volume ratio. A sensitivity increase of 57.4% was achieved in this experiment [108].

In order to reduce the cost of experiments, on the one hand, scientists have been exploring reusable experimental platforms; on the other hand, they have been exploring low-cost disposable experimental devices that can be mass-produced. In 2017, Feng et al. developed an optofluidic chip for the highly sensitive, label-free detection of 2,4-dichlorophenoxyacetic acid. The novelty of the optofluidic chip was the reusability based on the microring resonator. The experiment was completed with an LOD of 4.5 pg/mL [109]. In 2019, Tan et al. presented a fast and reproducible ELISA laser platform for the detection of interleukin-6 (IL-6). They sandwiched a top and a bottom mirror to form a microreactor with a high surface-to-volume ratio. As a result, they largely improved the repeatability and reliability of cavity mirror alignment [7]. Similarly, in 2020, Liu et al. developed a reusable optofluidic platform with lyophilized specific antibody for point-of-care-testing of cholylglycine in serum. They integrated evanescent wave fluorescence technology into an all-fiber-based optofluidic system to increase the reusability of the system. Although the LOD was 0.025 *μ*g/mL which was not enough for diagnostic criteria, the sensitivity could be improved simply by the dilution of the serum sample [110]. Different from the previous attempt to enhance reusability, in 2020, Yang et al. developed a low-cost disposable experimental device that could be mass-produced. This device was based on thin-wall hollow optical fibers (HOFs) which allowed the distribution of the identical laser microring resonators along the fibers. The reproducibility was validated with a low coefficient of variation of 3.3% [111].

In addition to the research on the improvement of sensitivity and low cost, scientists have also sought breakthroughs in integration. Before 2017, the reason why the practical implement of photonic biosensors within point-of-care platforms was difficult to realize was that the integration with fluidic automation subsystems was not easy. To solve this problem, Szydzik et al. created a lab-on-chip valve-based automation module, which helped fabricate normally closed pneumatically actuated elastomeric valves [112]. In 2018, Li et al. developed an integrated multichannel all-fiber optofluidic biosensing platform for the detection of atrazine and 2,4-dichlorophenoxyacetic acid (2,4-D). A 1 : 3 fiber optical switch and three single-multimode fiber optic couplers which greatly enhanced the integration of the entire system made up the M-AOB platform. This experiment was completed within 15 min with an LOD of 0.03 mg/L and 0.04 mg/L for atrazine and 2,4-D, respectively [113].

## 4. Conclusions and Future Perspectives

In this paper, the latest developments in microfluidic systems in immunoassays in the past decade have been reviewed in detail. Microfluidic immunoassay systems are used for disease diagnostic, environmental monitoring, and food and drug screening. According to different driving forces of fluid, the microfluidic platforms mentioned above are divided into two parts: passive manipulation and active manipulation. We expounded the principle, structure, performance, and improvement of every platform based on capillary-driven microfluidics, centrifugal microfluidics, electrophoresis microfluidics, optofluidics, magnetic microfluidics, and digital microfluidics, respectively. Compared with the traditional laboratory instruments, the performance of these microfluidic immunoassay systems is particularly excellent with no rise in the cost of mass production, which is good news for resource-limited areas.

However, there are still many difficulties for researchers to overcome. Firstly, most of the microfluidics using external pumps still have a large demand for power, which is not friendly to areas with power shortage. Secondly, although passive microfluidics avoids the trouble of using external pumps in active microfluidics, compared to active microfluidics, the control ability and accuracy of passive microfluidics are much inferior. Thirdly, when researchers focus on the miniaturization and low cost of the system, the functionality of the system may decline, which is an important issue that must be balanced. In the future, microfluidic immunoassay can also be combined with artificial intelligence, smartphone, 5G technology, and big data analysis to promote the development of POCT and provide the same medical resources for people in resource-limited areas.

## Figures and Tables

**Figure 1:** The classification of the different microfluidic platforms based on their driving force.

**Figure 2:** (a) The layout of the hollow-rivet-assisted movable valve paper device with open and closed conditions (reprinted with permission from [9], copyright 2017 AMER CHEMICAL SOC). (b) The three-dimensional fabrication of the capillary bead-based device with a chamber for packing beads (reprinted with permission from [10], copyright 2018 ELSEVIER SCIENCE SA). (c) Three-dimensional schematic diagram of the flow-through and the stopped-flow sePAD (reprinted with permission from [12], copyright 2019 AMER CHEMICAL SOC). (d) The layout of the microfluidic chip with its manipulation principles of the immunoassay (reprinted with permission from [13], copyright 2020 ROYAL SOC CHEMISTRY). MNPs: magnetic nanoparticles; QDs: quantum dots; CdTe: chitosan-coated.

**Figure 3:** (a) The illustration of the ZnO nanorod-decorated glass capillaries immunoassay (reprinted with permission from [14], copyright 2013 ROYAL SOC CHEMISTRY). (b) The flowchart of the transposition from a lateral flow assay to a microfluidic chip (reprinted with permission from [11], copyright 2020 AMER CHEMICAL SOC).

**Figure 4:** Schematic diagram of typical centrifugal microfluidic liquid propulsion (reprinted with permission from [23], copyright 2009 IEEE).

**Figure 5:** (a) Complete layout of a centrifugal microfluidic system with numbers indicating how a laser-irradiated ferrowax microvalve (LIFM) operates (reprinted with permission from [26], 2011 ROYAL SOC CHEMISTRY). TMB: tetramethylbenzidine. (b) Illustration of the principles of reciprocating flow and function image of speed changing with time (reprinted with permission from [27], 2011 AMER INST PHYSICS).

**Figure 6:** Frontal and lateral views layout of the structure of surface plasmon resonance (SPR) measurement disk with internal angle *θ*_int_ and externally measured angle *θ*_ext_ (reprinted with permission from [30], 2018 ELSEVIER ADVANCED TECHNOLOGY).

**Figure 7:** (a) The mechanism of elastic reversible (ER) valve (reprinted with permission from [32], 2019 ROYAL SOC CHEMISTRY). PMMA: polymethyl methacrylate; PSA: pressure-sensitive adhesive; PVC: polyvinyl chloride; PDMS: polydimethylsiloxane. (b) Illustration of the fabricated POC microfluidic immunoassay for procalcitonin detection (reprinted with permission from [34] 2018 MDPI). CAb: capture antibody; DAb: detection antibody; MAb: goat anti-mouse IgG antibody; FMS: fluorescent microspheres.

**Figure 8:** The layout of the working principle of pinch-valve. PMMA: polymethyl methacrylate; PDMS: polydimethylsiloxane. (a) The closed state of the system with flyball governor, actuation disc system, and microfluidic disc. (b) The open state of the system (reprinted with permission from [36] 2017, ELSEVIER SCIENCE SA).

**Figure 9:** (a) Flowchart of the operation step with a constant rotational speed setting (reprinted with permission from [38], 2018 ELSEVIER SCIENCE SA). (b) The 3D illustration of the Bento box with its internal structure and the block diagram of the motor control (reprinted with permission from [39], 2020 ROYAL SOC CHEMISTRY). (c) The schematic diagram of the system with patterned nitrocellulose membrane (a), patterned PMMA layer (b), the disc configuration (c), and the image of an assembled disc (d) included (reprinted with permission from [42], 2020 ROYAL SOC CHEMISTRY).

**Figure 10:** (a) The illustration of the layout of immunomagnetic detection platform with operation principle, microchannel dimensions, and schematic of the pneumatic flow system included (reprinted with permission from [52], 2011 ROYAL SOC CHEMISTRY). (b) The immunoassay format and dissolution process with photocurrent measurement (reprinted with permission from [54], 2017 AMER CHEMICAL SOC). MB: magnetic bead; PEC: photoelectrochemical; AFB1: aflatoxin B1; AFB1-BSA: AFB1-bovine serum albumin; CQDs: carbon quantum dots. (c) The three-dimensional illustration of the system with its and workflow chart (reprinted with permission from [60], 2020 PERGAMON-ELSEVIER SCIENCE LTD).

**Figure 11:** (a) The illustration of the immunoassay system with continual monitoring ability (reprinted with permission from [61], copyright 2016 NATURE PUBLISHING GROUP). (b) The illustration of the single-step magneto-immunoassay with spectrophotometric detection (a), electrochemical detection (b), and electrochemical detection at an MP-dsSPCE (reprinted with permission from [64], copyright 2020 ELSEVIER ADVANCED TECHNOLOGY). MP-dsSPCE: microfluidic paper, double-sided, screen-printed carbon electrode. (c) Illustration of the working principle for the integrated multicolor microfluidic immunoassay platform (reprinted with permission from [67], copyright 2020 AMER CHEMICAL SOC).

**Figure 12:** (a) Appearance of microfluidic chip and its micrograph of 30 analysis chambers for multiplexing detection (reprinted with permission from [71], copyright 2020 WILEY). (b) The illustration of the workflow of portable reusable accurate diagnostics with nanostar antennas (reprinted with permission from [72], copyright 2020 WILEY).

**Figure 13:** The illustration of the combination of the DMF with surface-enhanced Raman scattering-based immunoassay (reprinted with permission from [89], copyright 2018 AMER CHEMICAL SOC). DMF: digital microfluidic.

**Figure 14:** (a) An aptamer-based assay with the combination of a catalytic hybrid assembly and a microfluidic chip electrophoresis format, in which the reusable aptamer functionalized magnetic probes were used at room temperature (reprinted with permission from [100], copyright 2019 SPRINGER WIEN). APT: aptamer; CHA: catalyzed hairpin assembly; MC: microfluidic chip; FL: fluorescence; AFP: *α*-fetoprotein; CEA: carcinoembryonic antigen; CA125: carbohydrate antigen 125 (CA125). (b) The side view of the illustration of the immunoassay with nitrocellulose membrane (reprinted with permission from [101], copyright 2020 ROYAL SOC CHEMISTRY).

**Figure 15:** The illustration of optofluidic devices: (a) use a liquid-core arrow to trap particles and analyze fluorescence [105]; (b) the realization of parallel control for cells using optoelectronic tweezers (reprinted with permission from [105], copyright 2011 NATURE PUBLISHING GROUP). DMD: digital micromirror device; LED: light-emitting diode; AC: alternating current.

**Table 1:** Summary of typical capillary-driven microfluidic immunoassay platforms.

Improvement	Analyte	Performance	Characteristics	Reference
Valving innovation	CEA	LOD = 0.3 ng/mL	Movable valve to manipulate fluids	[9]
		Detection time = 60 min		

High integration	IgG	LOD = 1.7 ng/mL	Integrated microbeads and a no-wash, single-step mode	[10]

Step simplification	AFP	LOD = 0.63 ng/mL	Only a single introduction of a carrier buffer was needed	[12]
		Detection time = 30 min		

Step simplification	*Escherichia coli* and *Salmonella enteritidis*	LOD_1_ = 5 cfu/mL,	Only pipetting the samples and reagents was needed	[13]
		LOD_2_ = 3 cfu/mL		
		Detection time < 60 min		

High sensitivity	PSA, CEA, and AFP	LOD_1_ = 1 ng/mL,	Use ZnO nanorods to enhance fluorescent signals	[14]
		LOD_2_ = 5 ng/mL		
		LOD_3_ = 5 ng/mL		
		Detection time = 30 min		

Antibody immobilization	Rabbit IgG	LOD = 24.6 ng/mL	Immobilize capture antibodies in capillary-driven microfluidic chips	[15]
		Detection time = 20 min		

High sensitivity	rPfHRP2	LOD = 6 ng/mL	Combining sandwich immunoassays with electroless silver staining	[16]
		Detection time = 20 min		

High sensitivity	Cardiac marker troponin I	LOD = 4 ng/mL	Use self-coalescence modules and capillary assembled receptor carriers	[11]
		Detection time = 25 min		

High sensitivity	Anti-p53 autoantibody	LOD = 0.46 ng/mL	The system was in glass capillaries of 1 mm internal diameter	[17]
		Detection time = 45 min		

rPfHRP2, *Plasmodium falciparum* histidine-rich-protein 2; CEA, carcinoembryonic antigen; IgG, immunoglobulin; AFP, *α*-fetoprotein; PSA, prostate-specific antigen.

**Table 2:** Summary of the typical centrifugal microfluidic immunoassay platforms.

Improvement	Analyte	Performance	Characteristics	Reference
Mixing efficiency	Dengue NS1	Sample volume = 75 *μ*l	Centrifugal and capillary forces acted as a passive valve to control the flow sequence	[23]

Mixing efficiency	CHOL, HDL, TRIG, ALT, AST, GLU, and CKMB	Detection time = 22 min	Use silica beads with a larger mass	[26]

Mixing efficiency	Anti-goat IgG	LOD = 0.01 ng/mL	Reciprocating structure was combined with the pneumatic valve	[27]
		Detection time = 20 min		

Mixing efficiency	CRP	LOD = 4.9 pg/mL	Flow-enhanced electrochemical detection	[28]
		Detection time < 20 min		

Valving innovation	Hemoglobin A1c	SD = ±0.36%	A new passive valve, named septum valve, was used	[29]
		Detection time = 8 min		

Valving innovation	Human IgG	LOD = 19.8 ug/mL	Use the event-triggered valves with the CPSV	[30]
		Detection time < 60 min		

Multiplexing	CT, SEB, and SLT1	LOD_1_ = 2.02 ng/mL	Disposable disc with automatic aliquoting inlets was paired with a noncontact heating system	[31]
		LOD_2_ = 1.35 ng/mL		
		LOD_3_ = 5.5 ng/mL		
		Detection time < 60 min		

Multiplexing	Peptide arrays	Detection time = 40 min	Elastic reversible valves were used	[32]

Wash-free	CEA	LOD = 0.5 ng/mL	Use the effects of the medium density	[33]

Wash-free	Procalcitonin	LOD = 0.1 ng/mL	Use centrifugation step (15 s) to remove residual liquids and minimize nonspecific adsorption	[34]
		Detection time = 10 min		

High integration	Anti-mouse IgG	LOD = 1 ng/mL	Multiple layers of disk-like chips	[35]
		Detection time = 25 min		

High integration	Rabbit anti-mouse IgG	LOD = 20 ng/mL	A flyball governor and a group of spring plungers to form an integrated immunoassay system	[36]
		Detection time = 62 min		

High integration	Troponin T and NT-proBNP	LOD_1_ = 7.55 ng/mL	A disk-like microfluidic disposable cartridge contained all required dried and liquid reagents	[37]
		LOD_2_ = 16.566 ng/mL		
		Detection time = 11-12 min		

High integration	Human albumin	LOD = 0.707 ng/mL	It was designed on the principles of CLOCK	[38]
		Detection time = 18 min		

High integration	Mouse IgG	LOD = 0.32 ng/mL	A lab in a bento box made up of polypropylene	[39]
		Detection time = 12 min		

Highly automated	CRP	LOD = 1.5 ng/mL	Fully automated after the initial loading of sample and immunoreagents	[40]
		Detection time = 25 min		

Highly automated	CRP and interleukin 6	LOD_1_ = 1 ng/mL	Automation was controlled by the spinning frequency and without additional steps	[41]
		LOD_2_ = 64 pg/mL		
		Detection time = 30 min		

Highly automated	PSA	LOD = 0.028 ng/mL	Insert a nitrocellulose membrane into a centrifugal disc to obtain automation	[42]
		Detection time = 15 min		

CHOL, total cholesterol; HDL, high-density lipoprotein cholesterol; TRIG, triglycerides; ALT, alanine aminotransferase; AST, aspartate aminotransferase; GLU, glucose; CKMB, muscle and brain fraction of creatine kinase; CRP, C-reactive protein; SD, standard deviation; CPSV, centrifuge-pneumatic siphon valve; CT, cholera toxin; SEB, staphylococcal enterotoxin B; SLT1, Shiga-like toxin 1; CEA, carcinoembryonic antigen; CLOCK, control of liquid operation on centrifugal hydrokinetics; PSA, prostate-specific antigen.

**Table 3:** Summary of the typical magnetic microfluidic immunoassay platforms.

Improvement	Analyte	Performance	Characteristics	Reference
High sensitivity	Rabbit IgG and mouse IgG	LOD1 = 224 pg/mL	The specific applied magnetic field only moved the microbeads conjugated with superparamagnetic nanoparticles	[51]
		LOD2 = 15.4 ng/mL		
		Detection time = 35 min		

High sensitivity	CTC	25% less magnetic particles	The effective capture of labeled cells was achieved by the combination of the thin, flat dimension of the microchannel	[52]

High sensitivity	IL-17A	LOD = 0.05 ng/mL	The combination of magnetic Fe3O4@Au nanoparticles (GMNPs) and a magnetic field for an SPR immunoassay	[53]
		Detection time = 65 min		

High sensitivity	Aflatoxin B1	LOD = 2.1 pg/mL	Experiment was performed on anti-AFB1 antibody-modified magnetic beads	[54]
		Detection time = 15 min		

High sensitivity	PSA and PSMA	LOD1 = 15 fg/mL	A novel composite of Fe_3_O_4_ nanoparticles loaded onto graphene oxide (GO) nanosheets (Fe_3_O_4_@GO)	[55]
		LOD2 = 4.8 fg/mL		
		Detection time = 70 min		

High sensitivity	PSA	LOD = 0.31 pg/mL	Use reduced graphene oxide functionalized BiFeO_3_ (rGO-BiFeO_3_) as the photoactive material	[56]
		Detection time = 20 min		

High sensitivity	Superparamagnetic beads	LOD = 15 ug/mL	Use a magnetic frequency mixing technique with a set of miniaturized planar coils	[57]

High sensitivity	Aflatoxin B1	LOD = 3 pg/mL	Use OC-QDs and OAIONPs	[58]
		Detection time = 40 min		

High sensitivity	*Escherichia coli* O157 : H7	LOD = 50 cfu/mL	Use nanoparticle aggregation and smartphone as an imaging tool	[59]
		Detection time = 45 min		

High sensitivity	IL-6	LOD = 250 pg/mL	A chip-based scientific payload technology for visual detection	[60]

High integration	Transferrin	LOD = 0.03 ng/mL	Use disposable magnetic microbeads for immobilization and integrated microvalves	[61]
		Detection time = 75 min		

High integration	Thrombin	LOD = 25 pM	Apply an on-disc magnetic field-assisted incubation protocol	[62]
		Detection time = 15.5 min		

High integration	OTA, AFB1, and DON	LOD_1_ = 100 ng/mL	A novel, simple, negative pressure-driven device with manually operated magnetic valves	[63]
		LOD_2_ = 100 ng/mL		
		LOD_3_ = 3 ng/mL		
		Detection time < 20 min		

High integration	PfLDH	LOD = 2.47 ng/mL	The washing step, detection step, and filtration step were all conducted in an integrated disposable paper microfluidic device	[64]
		Detection time = 10 min		

Step simplification	PGA	LOD = 100 pg/mL	Use magnetic immunocomplexes trapped by yoke-type solenoids	[65]
		Detection time = 8–10 min		

Highly automated	Rabbit IgG	LOD = 1 pg/mL	Use bifunctional plasmonic magnetic nanoparticles to integrate micromixing and SERS detection	[66]
		Detection time = 80 min		

Highly automated	HIV-1 p24 antigen	LOD = 0.5 ng/mL	All the immunoreaction steps and the gold nanorod based assay were integrated into a single chip	[67]
		Detection time = 1.5 h		

Multiplexing	CEA and AFP	LOD_1_ = 0.01 ng/mL	Use biofunctionalized magnetic graphene nanosheets (MGO) as immunosensing probes and multifunctional nanogold hollow microspheres (GHS) as distinguishable signal tags	[68]
		LOD_2_ = 0.01 ng/mL		
		Detection time = 39 min		
Multiplexing	IL-6, IL-8, and VEGF	Range = 5–50 fg/mL	Beads were magnetically separated into the array when they finished the capturing of the proteins and the washing step	[69]
		Detection time = 50 min		

Multiplexing	Copeptin, h-FABP, and TnI	LOD_1_ = 0.4 ng/mL	Use magnetic carbon composites and a three-dimensional microfluidic paper-based device	[70]
		LOD_2_ = 0.32 ng/mL		
		LOD_3_ = 30.5 ng/mL		
		Detection time = 40 min		

Multiplexing	CTC	LOD = 1.5 ng/mL	Use the barcoded magnetic beads which were capable of CTC profiling	[71]
		Detection time = 65 min		

Multiplexing	cTnI and NPY	LOD_1_ = 0.005 ng/mL	Nanostar antennas were used	[72]
		LOD_2_ = 0.12 ng/mL		

Cost reduction	Glycated hemoglobin	LOD_1_ = 0.65 ng/dL	Use an aptamer-antibody assay on magnetic beads	[73]
		LOD_2_ = 8.8 g/dL		

Cost reduction	PSA	LOD = 0.01 ng/mL	Use magnetic pump	[74]
		Detection time = 5 min		

Cost reduction	HIV-1 and the p24 capsid antigen	LOD = 20 pg/mL	Syringe pumps or other peripherals to maintain the flow were not required	[75]
		Detection time = 20 min		

IL-17A, human interleukin 17A; CTC, circulating tumor cells; PSA, prostate-specific antigen; PSMA, prostate-specific membrane antigen; OAIONPs, oleic acid-modified iron oxide nanoparticles; OC-QDs, CdSe/ZnS QDs; OTA, ochratoxin A; AFB1, aflatoxin B1; DON, deoxynivalenol; PfLDH, plasmodium falciparum lactate dehydrogenase; PGA, poly-*γ*-D-glutamic acid; CEA, carcinoembryonic antigen; AFP, *α*-fetoprotein; IL-6, interleukin 6; IL-8, interleukin 8; VEGF, vascular endothelial growth factor; h-FABP, heart-type fatty acid-binding protein; cTnI, cardiac troponin I; CTC, circulating tumor cells; NPY, neuropeptide Y.
